The article "Concrete Application of Computer Virtual Image Technology in Modern Sports Training" was published in 2022. Journal: Comput Intell Neurosci.

# Concrete Application of Computer Virtual Image Technology in Modern Sports Training

**DOI:** 10.1155/2022/6807106

**Published:** 2022-03-08

**Authors:** YongHui Chi, Jun Li

**Affiliations:** ^1^Jilin University of Architecture and Technology, Changchun, Jilin Province 130114, China; ^2^Office of Teaching Construction and Quality Control, Chengdu Technological University, Chengdu, Sichuan Province 611730, China

## Abstract

The efficiency of basketball shooting training has always been an urgent problem to be solved in basketball sports. Applying computer virtual image technology to basketball sports training is the key to improve basketball shooting ability and improve the effect of basketball sports training. Therefore, based on the design of basketball shooting automatic recognition system based on the background difference method, this study puts forward the specific application of computer virtual image technology in modern sports training. By analyzing the techniques of image denoising, image detection, and image calibration, a goal detection algorithm for modern sports basketball shooting training is designed. Firstly, the camera is used for image capture, the RGB image is converted into gray image, and the median filter is used to suppress the noise in the image. Then, the background difference method is used to detect the moving region, and the background modeling is combined with the mean method. After obtaining the background reference model, the image is differentiated, the gray image after image difference is binarized, and then the binary image is postprocessed by morphological middle closure operation. Finally, the image calibration technology is used to extract the basketball feature information. Through the region segmentation algorithm, the basketball shooting part is segmented and judged, so as to realize the basketball shooting training goal detection. The experimental results show that the proposed method has a good effect on basketball shooting training goal detection and can effectively improve the detection accuracy and efficiency.

## 1. Introduction

The development of computer virtual image technology provides convenience for life. At present, computer virtual image technology is added to many devices in life [1–3]. With the rapid development of computer virtual image technology, moving target detection technology in video has been more and more widely used [4, 5]. Especially, in the application of modern sports training in recent years, the image processing technology in video includes image acquisition, processing, and image secondary display. Similarly, with the rapid development of the times, more and more requirements for video processing applications have been put forward. Moving target detection work is involved in many engineering application projects, but the moving target has a certain degree of difficulty in moving target detection due to the strong time-varying speed and uncertain path [6, 7]. Among them, the basketball special automatic test is an engineering application of sports target detection. The basketball special automatic test is one of the main content needed for the current sports professional basketball talent training test and basketball sports. Basketball goal recognition is the key technology of basketball special automatic test. Accurate and timely judgment of basketball goals has an important practical value.

The article "Concrete Application of Computer Virtual Image Technology in Modern Sports Training" was published in 2022. Journal: Comput Intell Neurosci.

At present, scholars in related fields have made some progress in basketball shooting detection. Yu and Liu [8] proposed an automatic feature detection method of the basketball shooting teaching image based on artificial intelligence. Starting from the decomposition of basketball shooting teaching actions, the practical attributes of basketball shooting teaching images are defined, and a standardized image detection environment based on artificial intelligence is constructed according to the essentials of basketball shooting actions. The feature of basketball shooting teaching image is extracted, the feature scale value of basketball shooting action is calculated, and the feature description principle of automatic detection is combined to complete the automatic detection of basketball shooting teaching image features. This method has certain validity. Yang et al. [9] proposed a three-dimensional multiviewpoint basketball player detection and location method based on probability occupancy. Combine player detection based on deep learning and player positioning based on occupancy rate to extract the characteristics of three-dimensional multiview basketball players. The Bayesian model of a new positioning algorithm is used to detect and locate basketball players' game images by using the foreground information of the fisheye camera. This method has high reliability.

Xie [10] designed an automatic shooting recognition system based on the background difference method. The design and application of the system are tested by experimental analysis, sampling survey, and data analysis. Firstly, the relevant information of the background difference method is collected, and the algorithm flow and modeling method of the background difference method are understood. Secondly, relevant tests are designed according to the characteristics of shooting. Then, an automatic recognition system is designed for experimental research. By sampling 8 basketball players for data observation and analysis, the results are obtained. The accuracy of the basketball shooting automatic recognition system reaches 89%, which can basically meet the requirements. Therefore, based on this research, this study puts forward the specific application of computer virtual image technology in modern sports training. Using computer virtual image technology, a goal detection algorithm for modern sports basketball shooting training is designed. The basketball shooting training images are captured and preprocessed, the background difference method is used to detect the motion area for background modeling, and the images are processed by difference and binarization before postprocessing. By extracting the basketball feature information, segmenting the basketball shooting part, and making judgments, the basketball shooting training goal detection is realized. The basketball shooting training goal detection effect of this method is better, and the detection accuracy and efficiency can be effectively improved.

The article "Concrete Application of Computer Virtual Image Technology in Modern Sports Training" was published in 2022. Journal: Comput Intell Neurosci.

## 2. Computer Virtual Image Technology

The number of virtual images from “brightest” to “darkest” is divided according to the gray level. The larger the dynamic range is, the richer the level can be represented and the wider the color space it contains. With the rapid development of computer technology, both software and hardware have developed to a very high level. However, for users who pursue higher quality, the development of computer is endless, especially, the requirements of image quality. In order to further improve the quality of some aspects of the virtual image and make it close to the real environment as much as possible, the computer virtual image technology is studied. The specific processing process is image denoising, image detection, and image calibration. The specific analysis is as follows.

### 2.1. Image Denoising Technology

Because the noise in different images has differences in characteristics and spectral distribution, different denoising methods are formed. The mean filtering method and the median filtering method are the two most typical denoising methods in the spatial domain.

#### 2.1.1. Mean Filtering Method

It uses the average brightness value or weighted value of all pixels in the neighborhood of gray jump points to replace the original jump pixel value, remove abnormal pixels, and realize image smoothing, so as to eliminate noise [11, 12]. The mathematical form of mean filtering is as follows:

(1) $$\begin{array}{c} g\left(x,y\right)=\frac{\sum_{i=1}^{mn}e_{i}d_{i}}{\sum_{i=1}^{mn}e_{i}}, \end{array}$$

where *d*_*i*_ is the neighboring pixel value of the jumping pixel *g*(*x*, *y*), *e*_*i*_ is the weighting coefficient of the neighboring pixel, that is, the template coefficient, and *mn* is the number of weighting coefficients, that is, the template size. If the neighborhood is larger, the image will be blurry accordingly. The average filter template is generally selected as the following size:

(2) $$\begin{array}{c} e=\frac{1}{9}\left[\begin{array}{ccc} 1 & 1 & 1\\ 1 & 1^{*} & 1\\ 1 & 1 & 1 \end{array}\right]. \end{array}$$

The position with an asterisk is the jumping pixel point, that is, the jumping point is at the center of the template. The equal weighting coefficient makes the pixels in the neighborhood play the same smoothing effect. Small amount of calculation and simplicity are the biggest characteristics of this filtering, but the smoothed image inevitably reduces the sharpness, especially the edges and details are the most obvious.

The article "Concrete Application of Computer Virtual Image Technology in Modern Sports Training" was published in 2022. Journal: Comput Intell Neurosci.

#### 2.1.2. Median Filter

It is a kind of the nonlinear smoothing filter, which can effectively suppress abrupt noise by using ranking statistical theory [13–15]. Working principles of the median filter are as follows: determine a pixel as the central position, sort the gray values of other surrounding pixels according to the size relationship, and take the intermediate value to replace the pixel value at the central position. A square neighborhood formed on the basis of the central pixel is called a window. The noise smoothing of the image is realized by moving the window. Median filtering algorithm can eliminate isolated noise points and reduce the fuzziness of the image.

In the one-dimensional case, if *b*_1_, *b*_2_, ..., *b*_*n*_ is a set of original signal sequences and assuming that *b*_1_, *b*_2_, ..., *b*_*n*_ is already an ordered sequence from large to small, then the median of this set of original signal sequences is defined as

(3) $$\begin{array}{c} k=median\left\{b_{1},b_{2},...,b_{n}\right\}=\left\{\begin{array}{c} b\left(\frac{n+1}{2}\right)\\ \frac{1}{2}\left(b_{\frac{n}{2}}+b_{\frac{n}{2}+1}\right) \end{array}\right\}. \end{array}$$

When there is a large isolated noise at the center of the slope change, the median filtering of this type of signal can completely eliminate the noise. When the noise is not isolated, but two consecutive equal values, the median filter can still completely filter out the noise in this case. At this point, the median filter has a much better effect than the neighborhood average smoothing.

In the two-dimensional case, the median filter takes the median value of the pixel gray value in the two-dimensional window as the new value at the center of the window, and its mathematical expression is

(4) $$\begin{array}{c} G\left(m,n\right)=median\left[f\left(i,j\right)\right] \end{array}$$

or

(5) $$\begin{array}{c} G\left(m,n\right)=median\left[f\left(m-i,n-j\right)\right]. \end{array}$$

Commonly used two-dimensional window shapes include cross window, X-shaped window, and square window. Commonly used processing windows for two-dimensional median filtering are shown in Figure 1.

The article "Concrete Application of Computer Virtual Image Technology in Modern Sports Training" was published in 2022. Journal: Comput Intell Neurosci.

### 2.2. Image Detection Technology

#### 2.2.1. Background Difference Method

The background difference method uses the difference between the pixel gray corresponding to the current frame image and the background image to detect the moving target [16–18]. The operation flow of the background difference method is shown in Figure 2.

Assuming that the background frame image used in the background difference method is static, that is, the background frame will not change with the number of image frames, *b*(*i*, *j*) is used to represent the background image, *μ*(*i*, *j*, *l*) is defined as the image sequence, and (*i*, *j*) in the image sequence is set as the position coordinate of the image. Among them, *l* is the number of frames in the image sequence, and the gray value of the selected image in the image sequence is used to make the difference with the gray value in the background image, and a difference image *μ*_*d*_(*i*, *j*, *l*) moving target is expressed as

(6) $$\begin{array}{c} \mu_{d}\left(i,j,l\right)=\mu \left(i,j,l\right)-b\left(i,j\right). \end{array}$$

#### 2.2.2. Interframe Difference Method

The interframe difference method is a method to obtain the contour of the moving target by frame difference between two consecutive frames extracted from video sequence [19–21]. The operation flow of the interframe difference method is shown in Figure 3.

The *τ* picture in the video sequence is recorded as frame *σ*, and the *τ* − 1 picture is regarded as frame *σ* − 1. The corresponding images are represented by *H*_*τ*_ and *H*_*τ*−1_, respectively, and the gray values of pixel points are represented by *H*_*τ*_(*i*, *j*) and *H*_*τ*−1_(*i*, *j*), respectively. The gray values of pixel points of two adjacent frames are subtracted to obtain the absolute value, and the two frames of differential images are expressed as

(7) $$\begin{array}{c} \kappa_{\tau }\left(i,j\right)=\left|H_{\tau }\left(i,j\right)-H_{\tau -1}\left(i,j\right)\right|. \end{array}$$

### 2.3. Image Calibration Technology

In order to obtain the size of the object and its corresponding position in the image from the video image, the relationship between the corresponding points in the object and the corresponding points in the image can be determined. The common method is image calibration technology [22–24]. The image calibration technology is divided into traditional camera calibration and camera self-calibration.

1. The traditional camera calibration method has certain requirements for the camera model, and the size and shape of the calibration object should be processed under the known condition. The internal and external parameters of the camera model can be obtained by mathematical transformation and calculation.
2. The camera self-calibration method does not require a specific calibration object, but is calibrated according to the positional relationship between the surrounding image and the corresponding image captured during the movement of the camera. Camera self-calibration methods can be further divided into camera automatic visual calibration technology, using basic matrix and essential matrix self-calibration technology, etc. Self-calibration technology is very flexible, but immature. Because there are too many unknowns, it is difficult to get stable results.

The article "Concrete Application of Computer Virtual Image Technology in Modern Sports Training" was published in 2022. Journal: Comput Intell Neurosci.

There are also differences in the selection of traditional camera calibration methods and camera self-calibration methods for different occasions. For example, for some occasions that require high accuracy and the parameters do not change frequently, traditional calibration techniques can be used. For communication, virtual reality, and other occasions where the accuracy is not high, the camera self-calibration method can be used.

## 3. Goal Detection Algorithm in Modern Sports Basketball Shooting Training

Through the further study of computer virtual image technology, this study puts forward the goal detection algorithm of modern sports basketball shooting training. The algorithm implementation flow is shown in Figure 4.

### 3.1. Image Capture and Preprocessing

In the process of basketball shooting training goal detection, the image capture position is very important. Whether the camera is installed properly directly affects the accuracy of detection. To this end, use the recorded TestOne video to detect and determine the installation position of the camera is set above the basket, and the camera installation position is directly opposite to the basket for image capture, which can completely capture the basketball goal process. Because the format of the video is RGB24, the color space parameters are not needed during the detection process, so after the image is acquired, the RGB image is converted to a grayscale image, thereby reducing the system memory usage and increasing the processing speed [25].

The image captured by the camera is easily disturbed and polluted by noise in the process of transmission, conversion, and storage, which will make the useful information in the image unable to be extracted. Therefore, after capturing and converting the image, this paper uses the median filter [26, 27] to suppress the noise in the image. In order to perform median filtering on a pixel point on an image, the pixel values of the desired pixel in the mask and its neighborhood must be sorted to determine the median, and the median is given to the pixel point, which is expressed as follows:

(8) $$\begin{array}{c} G\left(m,n\right)=media\left[f\left(m,n\right)\right]. \end{array}$$

The article "Concrete Application of Computer Virtual Image Technology in Modern Sports Training" was published in 2022. Journal: Comput Intell Neurosci.

### 3.2. Background Modeling

When using the background difference method to detect a moving area, the background reference model must first be prepared. Because the environment of the scene is relatively simple and the influence of other objective factors is small, this study adopts the mean value method for background modeling. The multiframe images captured by the camera in a period of time are accumulated, and then, the accumulated value is divided by the number of captured frames, and finally, the average value is obtained, and the obtained average value is used as the background reference model. The mathematical expression is expressed as

(9) $$\begin{array}{c} W_{n}=\frac{\left(z_{n}+z_{n-1}+...+z_{n-N+1}\right)}{N}, \end{array}$$

where *N* is the number of frames to be averaged, (*z*_*n*_+*z*_*n*−1_+...+*z*_*n*−*N*+1_) is the continuous *N* frame image saved by the system including the current frame, and *W*_*n*_ is the background model established by the system when the *n* frame image is collected. Due to the influence of the lighting changes in the scene and other factors and the background model updated according to the scene for a long time, it will cause the moving target to not be detected [28, 29]. Therefore, the obtained background model *W*_*n*_ must be updated at regular intervals, and the update calculation formula is

(10) $$\begin{array}{c} W_{n}=W_{n-1}+\frac{\left(z_{n}-z_{n-N}\right)}{N}. \end{array}$$

Formula (10) shows that the new background model is based on the background model *W*_*n*−1_ obtained in the previous calculation, and the current frame *z*_*n*_ and *z*_*n*−*N*_ frame are recursively obtained, thus realizing the update of the background model. Obviously, if the selected image frame *N* value (the more image frames) is larger, the background reference model *W*_*n*_ obtained is closer to the real background in the scene.

### 3.3. Image Difference

After the background modeling is completed, the foreground area is the area where the difference value of the current image minus the background image is greater than a specific threshold. Direct subtraction is generally good, but it is poor when the foreground and background are very similar, the noise is very loud, and there are shadows. At this time, the difference between the background area and the foreground area is relatively small, so it is difficult to select the threshold [30, 31]. For this reason, after the reference model is obtained, the image in the video can be differentiated to obtain the moving area in the image and separate the background in the image. For grayscale images, the following formula is used to perform differential operations indirectly:

(11) $$\begin{array}{c} \gamma \left(a,b\right)=1-\frac{2\sqrt{\left(a+1\right)\left(b+1\right)}}{\left(a+1\right)+\left(b+1\right)}\times \frac{2\sqrt{\left(256-a\right)\left(256-b\right)}}{\left(256-a\right)+\left(256-b\right)},\\ 0\leq \gamma \left(a,b\right)\leq 1,\\ 0\leq a\left(i,j\right),b\left(i,j\right)\leq 255, \end{array}$$

where *a*(*i*, *j*) and *b*(*i*, *j*) are the gray value of the current image and the background image at the pixel point (*i*, *j*), respectively. This formula can alleviate the impact of a particularly large or small pixel gray value.

The article "Concrete Application of Computer Virtual Image Technology in Modern Sports Training" was published in 2022. Journal: Comput Intell Neurosci.

### 3.4. Binarization Processing

After the image is differentiated, although some parameters of the image can be extracted, further processing of the image is required. In order to be able to quickly and accurately extract the position and appearance information of the basketball feature from the video image sequence, then it is necessary to binarize the gray image after image difference and to convert the gray image to binarization. First, a segmentation threshold value needs to be given, the gray value of the points in the grayscale image is compared with the given segmentation threshold value, and the grayscale image is converted into a binary image according to the result of the comparison. For this reason, the maximum interclass difference method [32, 33] is used to extract the threshold value in the grayscale difference image.

First, assume that the range of gray values in the entire image is [0, *L* − 1], and the number of pixels with gray values of *i* in the gray image is *c*_*i*_; then, *N* can be expressed as

(12) $$\begin{array}{c} N=\sum_{i=0}^{L-1}n_{i}. \end{array}$$

The occurrence probability of each gray value is

(13) $$\begin{array}{c} \sum_{i=0}^{L-1}m_{i}=1. \end{array}$$

The points in the grayscale image are divided into two regions *V*_0_ and *V*_1_ by the segmentation threshold *λ*. *V*_0_ is composed of points with grayscale value [0, *λ* − 1], and *V*_1_ is composed of points with grayscale value [*λ*, *L* − 1]. Then, the probabilities of regions *V*_0_ and *V*_1_ are, respectively,

(14) $$\begin{array}{c} M_{1}=\sum_{i=\lambda }^{L-1}m_{i}=1-M_{0},\\ M_{0}=\sum_{i=0}^{\lambda -1}m_{i}. \end{array}$$

The average gray levels of regions *V*_0_ and *V*_1_ are, respectively,

(15) $$\begin{array}{c} U_{0}=\frac{1}{M_{0}}\sum_{i=0}^{\lambda -1}m_{i}=\frac{U\left(\lambda \right)}{M_{0}}, \end{array}$$

(16) $$\begin{array}{c} U_{1}=\frac{1}{M_{1}}\sum_{i=\lambda }^{\lambda -1}m_{i}=\frac{U-U\left(\lambda \right)}{1-M_{0}}, \end{array}$$

where *U* is the average gray level of the entire image:

(17) $$\begin{array}{c} U=\sum_{i=0}^{L-1}m_{i}=\sum_{i=0}^{\lambda -1}m_{i}+\sum_{i=\lambda }^{L-1}m_{i}=M_{0}U_{0}+M_{1}U_{1}. \end{array}$$

The total variance of the two regions is

(18) $$\begin{array}{c} \omega_{B}^{2}=M_{0}M_{1}{\left(U_{0}-U_{1}\right)}^{2}. \end{array}$$

Let *λ* take values sequentially within the range of [0, *L* − 1] grayscale values so that the threshold *λ*, when the total variance *ω*_*B*_^2^ of the two regions is the largest, is the optimal region segmentation threshold in the grayscale image.

The article "Concrete Application of Computer Virtual Image Technology in Modern Sports Training" was published in 2022. Journal: Comput Intell Neurosci.

### 3.5. Mathematical Morphology Processing

After the gray image is processed by binarization, there will be many holes and gaps. In order to restore the basketball to its original shape and fill the hole, according to the effect of image difference and binarization, morphological closure operation [34–36] needs to be used for postprocessing of the binarized image. The closed operation can not only connect the disconnected adjacent targets in the binary image but also smooth the contour in the image.

First, the binary image is expanded, and then, the image is corroded. The definition is as follows:

(19) $$\begin{array}{c} \alpha \cdot \beta =\left(\alpha ⊕\beta \right)\Theta \beta , \end{array}$$

where *β* represents a structural element, *α* represents an image, and *α* · *β* represents *β* which performs a closed operation on the image *α*.

### 3.6. Basketball Feature Information Extraction

After the above steps and calculations and after the image is processed by mathematical morphology, the image calibration technology can be used to extract the basketball feature information. Basketball *x*_min_, *x*_max_*y*_min_, *y*_max_ is the minimum and maximum pixel coordinates in the *X*, *Y* direction, and it is also the basis for calculating other feature information. The total number of diameter pixels in the direction is denoted by *B*_*P*_(*X*)and*B*_*P*_(*Y*), and the calculation method is

(20) $$\begin{array}{c} \left\{\begin{array}{c} B_{P}\left(X\right)=x_{\max}-x_{\min}\\ B_{P}\left(Y\right)=y_{\max}-y_{\min} \end{array}\right\}. \end{array}$$

The corresponding pixel in the image and the actual corresponding size of the object are mainly obtained through the calculation of the calibration coefficient *B*_*T*_, which is a very important parameter in identifying goals, and the calculation of the basketball diameter is mainly obtained through *B*_*T*_. Only when *B*_*T*_ can be obtained accurately can we calculate some basketball parameters more accurately and judge basketball shots more accurately. In the image, a diameter line segment is marked in the basketball box, and two coordinate points (*x*_1_, *y*_1_)and(*x*_2_, *y*_2_) are obtained at both ends of the line segment. The total number of pixels *R*_*P*_ between the two points on the line segment can be obtained by the straight line calculation formula:

(21) $$\begin{array}{c} R_{P}=\sqrt{{\left(x_{2}-x_{1}\right)}^{2}+{\left(y_{2}-y_{1}\right)}^{2}}. \end{array}$$

The corresponding relationship between the length and the pixels established by the actual size of the basketball frame diameter *L* and the total number of pixels of the basketball frame diameter in the image is

(22) $$\begin{array}{c} B_{T}=\frac{L}{R_{P}}. \end{array}$$

Through the above extraction and calculation of basketball feature information, the basketball position can be determined.

The article "Concrete Application of Computer Virtual Image Technology in Modern Sports Training" was published in 2022. Journal: Comput Intell Neurosci.

### 3.7. Judging the Goal Method

The most important parameter for judging whether a basketball scores a goal is the actual size of the basketball diameter *B*_*R*_ in the image when the basketball is shooting:

(23) $$\begin{array}{c} B_{R}=\frac{B_{P}\left(X\right)+B_{P}\left(Y\right)}{2}B_{T}. \end{array}$$

The basketball shooting part is segmented by the area segmentation algorithm. When the basketball corresponding pixel is not detected in the basketball shooting and when the basketball shooting enters the basket, the total number of pixels in the *X*, *Y* direction of the basketball will be different. The ratio coefficient *Q* of the total number of pixels in this direction can be used to determine whether all basketball shots have entered the basket, which is expressed as

(24) $$\begin{array}{c} Q=\frac{B_{P}\left(X\right)}{B_{P}\left(Y\right)}. \end{array}$$

The method to judge the goal is to compare and analyze the eigenvalues of basketball calculated above. There are three conditions to judge whether a goal is scored. If any of the conditions are not met, it will be deemed that the basketball is not scored, and the image will be captured again for detection.

**Condition 1 .**

The calculated size of *B*_*P*_(*Y*) or *B*_*P*_(*X*) must be less than 24 cm. If it is larger than 25 cm, it means that the basketball is still above the ball frame and has not been put into the basketball frame.

**Condition 2 .**

Comparing *B*_*P*_(*Y*) and *B*_*P*_(*X*), if the ratio coefficient of the two is *Q* > 1.1 or *Q* < 1.1, it is possible to detect only the noise in the image or only a part of the basketball, indicating that the basketball is not all above the basket.

The article "Concrete Application of Computer Virtual Image Technology in Modern Sports Training" was published in 2022. Journal: Comput Intell Neurosci.

**Condition 3 .**

If the above two conditions are met, compare *B*_*R*_ with the diameter *B*_*T*_ of the basketball goal obtained in the debugging process. When *B*_*R*_ < *B*_*T*_, it is judged that the ball is scored, and *R*_*P*_ is automatically incremented by 1.

In the detection, the basketball shooting is judged through these three conditions. If the goal is judged, it will be delayed by 0.3 ms. This is because, after the goal, it is still possible to detect the basketball judged as after the goal. Then, the purpose of the delay is to wait for the previous one to pass through the basket, so as to avoid misjudgment. Through the above analysis, the computer virtual image technology is used to collect the basketball shooting image, and the image preprocessing is completed by establishing the background reference model, image difference, binarization processing, and mathematical morphology processing. On this basis, the basketball characteristic information is proposed and the goal determination method is designed to realize the basketball shooting goal detection in modern sports training.

## 4. Experimental Simulation and Analysis

### 4.1. Set up the Experimental Environment

In order to verify the effectiveness of the specific application of computer virtual image technology in modern sports training, simulation experiments are carried out in MATLAB. The operating environment is set in the GUIDE integrated environment of the MATLAB software GUI interface. In Intel Core i5-7200U@2.50 GHz CPU, 4G memory, Window 7 32 bit operating system, install this plug-in MCRInstaller.exe or MATLAB software and video decoder. In the process of basketball shooting, due to the fast movement of basketball, the basketball will hit the basket or backboard during the shooting process, causing the phenomenon of shooting jitter. For this reason, from the aspects of real-time, frame rate, and anti-shake, the camera model and CMOS sensor parameters are selected, as shown in Table 1.

### 4.2. Analysis of the Effect of Basketball Shooting Training Goal Detection

According to the above simulation environment and parameter settings, a basketball shooting training goal detection simulation experiment is carried out. Using the proposed method, through the recorded shooting video TestOne (640 × 480), the 46th, 85^th^, and 109th frames of basketball shooting training goal images are detected, and the basketball shooting training goal detection of the proposed method is obtained. The effect is shown in Figure 5.

According to Figure 5, the proposed method can effectively detect the basketball shooting training goal image, capture the goal track of the basketball shooting training image in frames 46, 85, and 109, and judge the basketball shooting training goal image. It can be seen that the basketball shooting training goal detection of the proposed method is better.

The article "Concrete Application of Computer Virtual Image Technology in Modern Sports Training" was published in 2022. Journal: Comput Intell Neurosci.

### 4.3. Analysis of the Accuracy of Goal Detection in Basketball Shooting Training

In order to further verify the basketball shooting training goal detection accuracy of the proposed method, the detection accuracy is taken as the evaluation index. The higher the detection accuracy is, the higher the detection accuracy is. The calculation formula is as follows:

(25) $$\begin{array}{c} A_{c}=\frac{P_{z}}{P_{j}}\times 100\%, \end{array}$$

where *P*_*z*_ represents the number of correctly detected goals and *P*_*j*_ represents the number of detected goals. The number of shots is set to 45. The methods of [8], the methods of [9], and the proposed methods are used to detect the basketball shooting training goal image, respectively. The comparison results of the detection accuracy of basketball shooting training goals of different methods are calculated according to formula (25), as shown in Figure 6.

It can be seen from Figure 6 that when the number of shots is 40, the average detection accuracy of basketball shooting training goals of the methods of [8] is 81.2%, the average detection accuracy of basketball shooting training goals of the methods of [9] is 74.5%, and the average detection accuracy of basketball shooting training goals of the proposed method is as high as 92.8%. It can be seen that the accuracy of basketball shooting training goal detection of the proposed method is high, which can effectively improve the accuracy of basketball shooting training goal detection. The main reason is that this method uses the background difference of the basketball shooting image in advance to improve the accuracy of basketball shooting training goal detection.

### 4.4. Analysis of the Efficiency of Goal Detection in Basketball Shooting Training

On this basis, the detection efficiency of the proposed method is verified. Taking the detection time as the evaluation index, the shorter the detection time, the higher the detection efficiency of the method. Using the methods of [8], the methods of [9], and the proposed methods, the basketball shooting training goal images are detected, and the comparison results of the detection efficiency of basketball shooting training goals of different methods are obtained, as shown in Figure 7.

It can be seen from Figure 7 that, with the continuous increase of shooting times, the goal detection time of basketball shooting training with different methods increases. When the number of shots reaches 45, the basketball shooting training goal detection time of the methods of [8] is 50 s and the basketball shooting training goal detection time of the methods of [9] is 37.5 s, while the basketball shooting training goal detection time of the proposed method is only 19.2 s. Therefore, the basketball shooting training goal detection time of the proposed method is short, which can effectively improve the basketball shooting training goal detection efficiency. The main reason is that this method accurately locates the goal position through image calibration, reduces the interference of background and other factors in the detection process, and improves the detection efficiency.

The article "Concrete Application of Computer Virtual Image Technology in Modern Sports Training" was published in 2022. Journal: Comput Intell Neurosci.

## 5. Conclusion

Taking basketball shooting training as the research object, this study completes the application research of computer virtual image technology in basketball shooting training from three aspects: image denoising, image detection, and image calibration. The experimental results show that this method gives full play to the advantages of computer virtual image technology, improves the accuracy and efficiency of goal detection in modern sports basketball shooting training, and has a good effect of goal detection in basketball shooting training. However, this method is only applied in basketball shooting training goal detection. The next research is to apply and analyze it in other aspects of basketball training or other sports, expand the algorithm, and further improve the application universality of the proposed method.

## Figures and Tables

**Figure 1:** Common processing windows for two-dimensional median filtering.

**Figure 2:** Background difference method operation flowchart.

**Figure 3:** Interframe difference method operation flowchart.

**Figure 4:** Algorithm implementation flowchart.

**Figure 5:** Basketball shooting training goal detection effect of the proposed method.

**Figure 6:** Comparison results of goal detection accuracy of basketball shooting training with different methods.

**Figure 7:** Comparison results of goal detection efficiency of basketball shooting training with different methods.

**Table 1:** Set model parameters.

Project	Model	Free drive (M30 A)
Video camera	Image resolution	640 × 480
	Frame rate	60 frames/sec
	Interface protocol	USB2.0
	Image data format	YUV422
	Programmable control	Brightness, contrast, hue, saturation, etc.
CMOS sensor	Pixel size	6 × 6 *μ*m
	Photosensitive size	3984 × 2953 *μ*m
	Sensitivity	3.0 V/Lux-sec (550 nm)
	Spectral response	310–1070 nm affixed IR650 filter

## Data Availability

The raw data used to support the findings of the study can be obtained from the corresponding author upon request.
